# Quantitative Measurements of the Depth of Enamel Demineralization before and after Bleach: An In Vitro Study

**DOI:** 10.1155/2022/2805343

**Published:** 2022-08-27

**Authors:** Sara Naim, Gianrico Spagnuolo, Essam Osman, Syed Sarosh Mahdi, Gopi Battineni, Syed Saad B. Qasim, Mariangela Cernera, Hasna Rifai, Nada Jaafar, Elie Maalouf, Carina Mehanna Zogheib

**Affiliations:** ^1^Department of Esthetic and Restorative Dentistry, Saint Joseph University of Beirut, Lebanon; ^2^Department of Neurosciences, Reproductive and Odontostomatological Sciences, University of Naples “Federico II”, 80131 Napoli, Italy; ^3^Beirut Arab University, Beirut, Lebanon; ^4^Dental Section of Jinnah Medical and Dental College, Sohail University, Karachi, Pakistan; ^5^Centre of Clinical Research, School of Medicinal and Health Products Sciences, University of Camerino, Camerino, Italy; ^6^Department of Bioclinical Sciences, Faculty of Dentistry, Kuwait University, Kuwait City, Kuwait; ^7^Department of Pediatrics, School of Dental Medicine, Lebanese University, Beirut, Lebanon; ^8^Department of Periodontology, School of Dental Medicine, Lebanese University, Lebanon; ^9^Department of Esthetic and Restorative Dentistry, Faculty of Dental Medicine, Saint Joseph University of Beirut, Lebanon

## Abstract

**Objective:**

This study is aimed at determining two main points. First, if the Canary System™ (CS), initially used to assess caries, can measure a decalcification depth of bleached enamel quantitatively, and second, whether or not whitening has a harmful effect on enamel. This device can be considered a useful tool in the clinical assessment of the progression of demineralization after bleaching.

**Materials and Methods:**

This study collected sixty human premolars that are in a good state recently extracted for orthodontic reason. To properly disinfect and preserve the premolars, they were stored in a saline solution and later in distilled water for a period of two weeks to allow the premolars to rehydrate. Later, 24 hours before the experiment, the premolars were introduced into a solution of artificial saliva to acquire back their minerals. The mineral content of the teeth was measured by the Canary System™ before bleaching. The teeth were bleached with 30% hydrogen peroxide (fläsh HP 30%), 30 min per week and for 3 consecutive weeks to simulate the conditions of strong bleaching in the clinic. The extent of demineralized enamel was measured by the Canary System™ at three points on the enamel surface of each tooth. The data were averaged for each application of the bleaching product. The demineralization extent of the teeth was measured by the Canary System™ before and after bleaching. The significance level was set at 0.05, and SPSS version 26 was used. The data were analyzed by using Wilcoxon's and Student's tests.

**Results:**

Mineral loss occurred after the first bleaching session; the Canary System™ detected a decalcification in the first bleaching session (532 ± 322 *μ*m) compared to the other sessions (*p* ≤ 0.05), while no significant change was detected between the second and the third sessions (*p* > 0.05).

**Conclusion:**

Based on the findings of the present study, under in vitro conditions, it was possible to measure the demineralization extent of bleached enamel with the Canary System™.

## 1. Introduction

With the increasing demand for well-aligned teeth and beautiful smiles, dental cosmetic treatments have become highly demanded. In this context, teeth bleaching is one of the top wishes of patients looking for a beautiful smile [1]. Compared to other bleaching processes, bleaching is considered to be the most conservative treatment as it preserves the tissues [2, 3]. Bleaching techniques may be classified by whether they involve vital or nonvital teeth and by whether the procedure is performed in the office or at home. The most popular technique is the in-office bleaching that involves 35% hydrogen peroxide; it is found to be a more reliable option [3], because it is totally under the dentist's control, and the soft tissue is generally protected from the process and has the potential for bleaching quickly. In the early stages of in-office bleaching treatment, 8%-66% of patients experience a moderate degree of teeth sensitivity [4, 5].

As a process, the bleaching treatment involves the application of a bleaching gel to the surface of the tooth for a short period. This application, however, would adversely affect the enamel structure in a way that would lead to teeth sensitivity due to increased porosity of the enamel. As a result, the bleaching gel would penetrate the dentin through the dentinal tubules and even into the dental pulp. Hence, changing the microhardness of the enamel and increasing roughness of the enamel surface [6]. Bleaching treatment can cause some side effects such as dentin hypersensitivity, gingival irritation, alteration of tooth surface morphology, and dehydration [7]. There have been several discussions concerned about the enamel microhardness, before and after bleaching procedure, and the subsequent works on this topic have established diverse results. According to studies [8, 9], enamel microhardness is associated with demineralization and has been measured by Vickers, a conventional measurement tool. However, there is no indication that the demineralization of enamel has been measured by a corresponding mineral measuring instrument. As the main mineral salts constituting the enamel are calcium and phosphorus, demineralization is effectively the leakage of these minerals from the mineralized tissues due to acid dissolution.

The Canary System™ is a noninvasive device that enables the early detection of dental caries. The caries process is a dynamic phenomenon that follows large fluctuations in pH in the biofilm on the surface of the teeth. Clinically, the affected area will become “sticky” or “soft” on probing and will show visual signs of demineralization. Accordingly, a lesion of 10 to 15 microns develops below the surface of the teeth while the surface layer is intact and could not be probed during the early stages of its formation. Nevertheless, continuous acid diffusion will ultimately lead to increased demineralization of subsurface enamel. Subsequently, this will cause further decalcification to a level reaching below the intact surface layer [10]. In the case of a 50-micron lesion, the Canary System™ can measure up to 5 mm in diameter below the tooth surface [11]

Lesion severity is expressed by the Canary System on a scale of 0-100 [12, 13]. The Canary System™ uses photothermal radiometry and luminescence (PTR-LUM) to explore the crystal structure of the tooth. This is achieved by measuring the heat and the light that are converted from the surface of the tooth when laser hits it. The PTR-LUM may perform various functions, including but not limited to examining sites suspected of ‘hidden caries,' obtaining an estimate of how severe the lesion is in depth and extent. The results is provided in terms of canary numbers to assist in better decision making when it comes to treatment, measuring and recording the initial quantitative value of demineralization and allowing quantitative monitoring of the evolution of lesion activities such as the progression of demineralization overtime during nonoperative management. According to Abrams et al., the Canary System™ uses a complex algorithm [14] that converts PTR/LUM signals to canary numbers using a scale from 0 to 100 that appears on a monitor screen. In particular, the system classifies the characteristics of both the signal strength and the depth of the tooth into three zones: healthy zone, zone with deterioration, and zone with advanced deterioration. Each of these zones is characterized with a specific range. For instance, a healthy zone has a canary number that ranges from 0 to 20 indicating that there is no decalcification. The zone with deterioration has a canary number that ranges from 21 to 70, indicating that the decalcification is as deep as (532 ± 322 *μ*m). As for the third zone, the zone with advanced deterioration, the canary number ranges from 71 to 100, indicating that the decalcification is as deep as (1057 ± 441 *μ*m).

The measurement of demineralization would facilitate the assessment of the mineral content of the tissues as well as whether there has been a loss of minerals because of the dissolution of the inorganic part, likewise what takes place during a caries process. In addition, such measurement would assist with quantifying the gain in density using an ion incorporation process (remineralization). Accordingly, the Canary System™ should be very efficient in performing these measurements due to its high sensitivity in detecting caries and dental decalcification also called demineralization when the enamel loses its minerals and erodes.

Based on the abovementioned overview, this study is aimed at determining two main points. First, to measure quantitatively the demineralization extent of bleached enamel by using a new quantitative device of measurement: the Canary System™, and the second aim was to determine whether teeth bleaching has a detrimental effect on enamel.

The null hypotheses were as follows:

- The first null hypothesis: the Canary System™ cannot measure decalcification before and after bleaching
- The second null hypothesis: there is no change in the mineral content of the enamel before and after in office bleaching with 30% of HP
- The third null hypothesis: saliva does not play a role in the recovery of mineral constituents of enamel

## 2. Methods

The Ethics Committee of “Saint Joseph” University of Beirut has reviewed and approved the protocol of this study under the number USJ-2021-163.

### 2.1. Specimens

In this experimental study, 60 healthy recently extracted human premolars were collected and conserved in saline solution to disinfect the teeth and to keep them well-preserved. Healthy freshly extracted human premolars for orthodontic treatment with full roots were only included in this study since premolars are easy to be collected and are included in office bleaching.

The roots of the teeth were mounted in cylindrical acrylic resin blocks (1.5 × 2.5 cm), with only the coronal part of the tooth (above the enamel junction) out of the block (Figure 1).

The device was calibrated following the instructions of the manufacturer's user manual. Using Quick Scan setting in the device, the scans of the Canary System were applied after ensuring that the study site is dry. The tip of the device was moved to three points of the buccal surface of the enamel. The teeth were provided with distinct numbers to distinguish which teeth are healthy and which had damaged surfaces. Accordingly, healthy teeth had values ranging from zero to 20, while teeth with a damaged surface had values greater than 20. (Figure 2).

### 2.2. Treatment Procedures

In an attempt to approach the clinical conditions, the bleaching procedures were preceded by teeth polishing, the buccal enamel surfaces under experimentation were polished with a Robinson brush and prophylactic paste [15] (Cleanic, KerrHawe SA, Via Strecce, CH-6934 Bioggio).

In an ultrasonic bath which contained distilled water, the teeth were placed for 10 minutes at different phases: between each polishing step and at the end of the polishing procedure. This is critical in order to remove the residual particles of polishing paste before storing the teeth in distilled water for a period of two weeks. Throughout the two weeks period,the teeth will be rehydrated, [16]. Next, the teeth were dried out and the demineralization extent of each tooth was measured by the Canary System™ at three points on the buccal surface of the enamel and the data were averaged [17].

24 hours before the experiment, all teeth were stored in artificial saliva (*Biotène* Dry Mouth Oral Rinse, MoonTownship*, PA,* USA) containing water, glycerin, xylitol, sorbitol, propylene glycol, poloxamer 407, sodium benzoate, hydroxyethyl cellulose, methylparaben, propylparaben, flavor, sodium phosphate, disodium phosphate with a pH between 6 and 7.8, and the demineralization extent of each tooth was measured at three points of the buccal surface of the enamel and the data were averaged. Then, the teeth were bleached with 30% hydrogen peroxide (fläsh; WHITEsmile, Germany) for 30 min per week and for three consecutive weeks to simulate the strong bleaching conditions in the clinic (Figure 3). The bleaching agent was rinsed under running water for one minute; then, the teeth were dried out, and the demineralization extent was measured by the Canary System™ at three points of the buccal enamel surface, and the data was recorded and averaged; then, the teeth were kept in a remineralizing solution (artificial saliva).

Finally, an average of three readings was recorded and this average was used for statistical analysis.

### 2.3. Statistical Analysis

SPSS V26 was used to conduct statistical data analysis, and the significance level was set at 0.05. The sample was more than 30, the Kolmogorov-Smirnov test could have been skipped but to ensure the normality of distribution of variables at the level of the teeth, and this test was used. To evaluate the change in the mineral content of the teeth, before and after applying the bleaching product, the Student test (parametric test) was adopted. However, to compare the mineral content before and after applying the bleaching treatment, the Wilcoxon test (nonparametric test) was adopted. The condition to paired *t*-test was not assumed, and we had a paired samples that why we used a nonparametric test.

## 3. Results

60 recently extracted healthy human premolars were analyzed. After storing the teeth in distilled water at 37°C for 24 hours, the average of the 3 values of the canary number was of the order of 21.8 ± 4.6 with a minimum value of 15 and a maximum of 35.6. Subsequently, storing the 60 teeth in a remineralizing solution (artificial saliva), the average of the three values of the canary number was of the order of 14.3 ± 1.5 with a minimum value of 11 and a maximum of 16.6, indicating all the teeth were healthy. After the three subsequent bleaching sessions, the average of the three values of the canary number was of the order of 23.8 ± 4.5, 18.3 ± 3.5, and 18.04 ± 3.12, respectively. The presence of a loss of minerals indicates that there were teeth that showed areas of deterioration with a decalcification depth of 532 ± 322 *μ*m in three sessions.

Table 1 presents the statistical analysis of sound and bleached enamels with 30% of HP fläsh.

The comparison of the percentages of healthy teeth before and after bleaching is depicted in Figure 4. After storage in distilled water, 31 teeth (51.7%) were considered healthy and 29 (48.3%) decalcified. After storing them in a remineralizing solution, all the teeth became healthy. While comparing the three bleach sessions, the final session was produced 85% (*N* = 51) of healthy teeth and a low percentage of demineralized teeth Table 2.

Table 3 presents the *p* value estimations of Students' tests.

The depth of enamel decalcification (or mineral loss) of teeth stored in distilled water was significantly different from the depth of enamel decalcification when teeth were stored in saliva (*p* < 0.001). The depth of enamel decalicification when teeth were stored in the saliva was significantly different from the depth of enamel decalcification obtained after all bleaching sessions (*p* < 0.001). However, there was no significant difference between the second and the third whitening session (*p* = 0.536).

Based on our study outcomes, a 30% hydrogen peroxide solution demineralizes enamel. Moreover, enamel measurements revealed a reduction in the levels of calcium (Ca) and phosphorus (P). Hence, the bleaching agents has resulted in the reduction of these mineral elements from teeth. Based on our results, demineralization occurred after the first bleaching session. The Canary System™ detected a depth of decalcification of 532 ± 322 *μ*m which corresponds to enamel mineral loss compared to the other sessions (*p* ≤ 0.05), while no significant change was detected between the second and the third sessions (*p* > 0.05).

## 4. Discussion

According to the results of this study, the three null hypotheses were rejected: the CS was able to measure the demineralization between the baseline and after bleaching, there was a statistically significant demineralization of the enamel surface, and the saliva played an important role in remineralization of enamel.

This study is aimed at quantitatively assessing the depth of enamel decalcification or the volume of mineral loss that can occur in patients who undergo strong bleaching in the clinic via a mineral measurement system which is the Canary System™. It is critical to highlight that the Canary System™ allows for specific measurement of the crystal structure of a tooth. Specifically, the Canary System ™ measures across 0.5 microns in diameter and up to 5 mm in depth. As a result, the Canary System™ uses a scale of 0-100 to indicate the state of the enamel's crystal structure. This number, however, accounts for both the volume of the demineralized tissue, as well as the depth of the lesion [18].

Another indication of the loss of minerals in the teeth is the surface microhardness of the enamel and the dentin. By definition, surface microhardness of a tooth helps in determining the mechanical properties of both, the surface of an enamel and the dentin. These properties are linked to the level of loss or gain of minerals within the crystal structure of the tooth [19]. Regardless of the pH of the bleaching gel, the mineral loss after bleaching and the alteration of the enamel structure are due to the breakdown of hydrogen peroxide found in the whitening gel into highly reactive radicals [20].

Based on studies on demineralization, when the enamel undergoes a demineralization as a result of bleaching, the superficial microhardness decreases without returning to its original values. This takes place irrespective of the pH level of the bleaching agent [21–24]. Clinically, it is demonstrated that enamel loss of calcium and phosphorous minerals can be prevented [25]. The parotid gland secretes urea, and this secretion may help boost the flow of saliva, hence enhancing the basic nature of the oral cavity. Because of the oral cavity becoming more basic, the enamel demineralization process is hindered [25]. This study showed that after the second and third sessions of bleaching, no significant difference was observed in the decalcification of the enamel surface. Accordingly, the saliva played a critical role in the recovery of the enamel microhardness postbleaching, as well as remineralizing the enamel (refer to Table 3). Moreover, the salivary proteins helped accumulate calcium and phosphate precipitations inside the enamel. This resulted in the enamel returning to its normal state after sometime [26].

According to Li et al. [27], 38% of HP bleaching treatment led to demineralization of the outer layer. Our results concur with those previous ones reporting that bleaching application results in demineralization and that the loss of mineral ions can be controlled naturally through the saliva. Regarding the change in the number of healthy teeth before and after bleaching, after storage in distilled water, they were considered healthy. After storing them in a remineralizing solution, all the teeth became healthy. Another literature study [28] supports our results in concluding that the demineralization process of the enamel microhardness; as a result of changes in HP, it can be reversed by the ability of saliva to remineralize the enamel, hence providing it with the calcium and phosphate ions lost in the bleaching process.

According to Grazioli et al. [29], enamel can be remineralized within 14 days after bleaching, as a result of the calcium and phosphate concentrations in the saliva. Specimens had regained their microhardness within two weeks following bleaching with HP based gel of a neutral pH [30]. Based on the results of the statistical analysis of the study, our results showed that demineralization occurred (532 ± 322 *μ*m) only in the first bleaching session compared to the other sessions (*p* < 0.05), which corresponds to enamel mineral loss while there was no significant change between the second and the third sessions. It would be interesting to analyze the mineral makeup of this new layer and see if further applications of HP could demineralize it.

This concludes that superficial mineral loss may occur only in the first session of the specimen of 30 min bleaching with 30% of hydrogen peroxide and the saliva can remineralize teeth and may inhibit the demineralization process between the second and the third session. The results of this study confirm what the literature exhibited [31, 32]; when compared to other bleaching sessions, all teeth have regained their minerals seven days after bleaching and after being stored in the artificial saliva.

Nevertheless, other studies concerning the demineralization and the microhardness of thinned enamel, before and after bleaching, have been controversial, and diversity of results has been obtained in the different works carried out. Some studies did not result in changes to the enamel surface after bleaching, nor was there change to the topography of enamel and dentin [33–35]. These studies concluded that despite using high concentrations of HP, the enamel was preserved.

These contradictory results may be attributed to several differences in the approaches adopted in the studies. Such differences might relate to adopting a different methodology than the one adopted in this study. For example, these studies might have used different bleaching agents or microhardness evaluation mechanisms or pH level or storage method of the specimens [36].

Bleaching is a viable alternative treatment to attempt aesthetic improvement of discolored teeth. Depending on the type and the severity of tooth discoloration, the tooth can be treated by bleaching, veneering, or a combination of both [37].

Bleaching is considered before porcelain veneer placement to either eliminate the need for veneers, reduce the amount of opacifiers needed to mask discoloration, or to give the patient the option of attempting a less expensive invasive treatment before committing to veneers [38].

Full-coverage restoration are one of the most popular and versatile options other than veneers but they are not a conservative treatment. There are also other alternatives to in-office bleaching like resine composite veneers. It is more affordable than porcelain veneers, and it is used to improve the appearance of a discolored tooth when bleaching fails to treat the discoloration [39]. However, direct resine composite veneers have some disadvantages like color stability, less resistance against abrasions, and fractures [40].

Previous studies have shown that bleaching agents affect the microtensile bond strength (*μ*TBS) of a composite to the enamel due to oxygen liberation during the bleaching process [41–43]. The main cause of this reduction is the presence of residual oxygen in the enamel and dentin which prevents the infiltration of the adhesive into the etched enamel or partially inhibits its polymerization. To overcome this problem and restore immediately the bond strength between the composite and the bleached enamel, applying 10% of sodium ascorbate (SA) for 10 min is the solution [44]. This method is a clinical alternative for patients in need of immediate aesthetic restoration after bleaching [39].

The literature and this study both confirm that saliva plays a critical role in remineralizing enamel that have been bleached.

The limitations of this study were as follows:

- The study was carried out in vitro, and therefore, we could not perfectly mimic the oral conditions
- A small sample size can affect the outcome significantly
- Using one concentration of HP with acidic pH does not help extrapolate the results to other concentrations and pHs
- The Canary System™ may be influenced by the thickness of the enamel

## 5. Conclusions

Based on our findings, under in vitro conditions, it was possible to measure the demineralization of bleached enamel with the Canary System™. Despite the need to further explore the level of accuracy of the Canary System, our findings showed that the Canary System™ was able to measure a decalcification of bleached enamel. Hence, and within the limitation of this study, the Canary System™ could be considered a relevant and reliable tool for clinically assessing the progression of demineralization after bleaching. Additionally, our findings conclude that teeth lose minerals when treated with 30% hydrogen peroxide; however, the damaging effect does not last long. Further clinical trials are recommended to validate this conclusion.

## Figures and Tables

**Figure 1:** Teeth mounted in cylindrical acrylic resin blocks.

**Figure 2:** Enamel demineralization measurement.

**Figure 3:** Bleaching buccal surface of enamel (fläsh 30% HP).

**Figure 4:** Comparison of the percentages of healthy teeth before and after bleaching.

**Table 1:** Mean and standard deviation of sound enamel and bleached enamel (*N* = 60).

	Distilled water	Saliva	First session	Second session	Third session
Mean	21.81	14.2	23.81	18.37	18.04
SD	4.64	1.5	4.52	3.50	3.12

**Table 2:** Number of healthy teeth before and after bleaching.

	Sound teeth			Demineralized teeth		
	*N*	%	*m* ± sd (*μ*m)	*N*	%	*m* ± sd (*μ*m)
Distilled water	31	51.7	18.63 ± 1.86	29	48.3	25.21 ± 4.32
Saliva	60	100	14.26 ± 1.50	0		
First session	19	31.7	18.26 ± 1.80	41	68.3	26.38 ± 2.71
Second session	50	83.3	17.16 ± 2.1	10	16.7	24.45 ± 2.70
Third session	51	85.0	17.96 ± 3.47	9	15.0	20.71 ± 2.83

**Table 3:** *p* value estimated from Student's test.

	Saliva	First session	Second session	Third session
Distilled water	<0.001	0.006	<0.001	<0.001
Saliva		<0.001	<0.001	<0.001
First session			<0.001	<0.001
Second session				0.536

## Data Availability

Readers can access the data used in this work by sending special requests to the Saint Joseph University of Beirut.
